The article "Computerized Tomography Image Features under the Reconstruction Algorithm in the Evaluation of the Effect of Ropivacaine Combined with Dexamethasone and Dexmedetomidine on Assisted Thoracoscopic Lobectomy" was published in 2021. Journal: J Healthc Eng.

# Computerized Tomography Image Features under the Reconstruction Algorithm in the Evaluation of the Effect of Ropivacaine Combined with Dexamethasone and Dexmedetomidine on Assisted Thoracoscopic Lobectomy

**DOI:** 10.1155/2021/4658398

**Published:** 2021-11-10

**Authors:** Yan Cui, Yang Sun, Meng Xia, Dan Yao, Jun Lei

**Affiliations:** ^1^Department of Anaesthesia, Affiliated Nanjing Brain Hospital, Nanjing Medical University, Nanjing 210029, China; ^2^Department of Anaesthesia, Nanjing Chest Hospital, Nanjing 210029, China

## Abstract

This research was aimed to study CT image features based on the backprojection filtering reconstruction algorithm and evaluate the effect of ropivacaine combined with dexamethasone and dexmedetomidine on assisted thoracoscopic lobectomy to provide reference for clinical diagnosis. A total of 110 patients undergoing laparoscopic resection were selected as the study subjects. Anesthesia induction and nerve block were performed with ropivacaine combined with dexamethasone and dexmedetomidine before surgery, and chest CT scan was performed. The backprojection image reconstruction algorithm was constructed and applied to patient CT images for reconstruction processing. The results showed that when the overlapping step size was 16 and the block size was 32 × 32, the running time of the algorithm was the shortest. The resolution and sharpness of reconstructed images were better than the Fourier transform analytical method and iterative reconstruction algorithm. The detection rates of lung nodules smaller than 6 mm and 6–30 mm (92.35% and 95.44%) were significantly higher than those of the Fourier transform analytical method and iterative reconstruction algorithm (90.98% and 87.53%; 88.32% and 90.87%) (*P* < 0.05). After anesthesia induction and lobectomy with ropivacaine combined with dexamethasone and dexmedetomidine, the visual analogue scale (VAS) decreased with postoperative time. The VAS score decreased to a lower level (1.76 ± 0.54) after five days. In summary, ropivacaine combined with dexamethasone and dexmedetomidine had better sedation and analgesia effects in patients with thoracoscopic lobectomy. CT images based on backprojection reconstruction algorithm had a high recognition accuracy for lung lesions.

## 1. Introduction

Lobectomy is mainly used for malignancies confined to the lobes, lung damage caused by tuberculosis, severe bullae, bronchiectasis, interstitial lesions, trauma, and dysplasia, which refers to routine removal of the lungs [1]. There are five lobes in the chest. The right lung is made up of the upper, middle, and lower lobes. The left lung is made up of two lobes, the upper and lower lobes. Lobectomy is used for lung cancer and irreversible disease confined to the lung lobe. It mainly includes right upper lobe resection, right middle lobe resection, right lower lobe resection, left upper lobe resection, and left lower lobe resection. If the lesion involves both lobes or intermediate bronchial tubes, upper middle or lower middle lobe pneumonectomy is feasible [2]. In general, the postoperative quality of life of patients is not bad. Postoperative patients need to pay attention to the change of climate and pay attention to diet and avoid irritant gases in normal survival [3]. In addition, it is necessary to take proper exercise to strengthen resistance and closely observe the symptoms and signs of oneself. If abnormal, it is necessary to go to the hospital for comprehensive examination and treatment as soon as possible [4, 5]. Thoracoscopic lobectomy is a kind of lobectomy in which the thoracoscopic surgeon only watches the thoracoscopic situation through the TV screen in real time and performs the operation through one to four hole-like incisions no longer than 5 cm (without repositioning the ribs). Veins, arteries, and bronchial tubes were dissected anatomically, and the lung lobe was completely removed. At present, video-assisted thoracic surgery (VATS) lobectomy is basically mature and widely accepted. Its surgical techniques are also gradually refined and improved [6, 7]. The National Comprehensive Cancer Network (NCCN) guidelines for the treatment of lung cancer clearly state that “VATS lobectomy is a viable option for resectable lung cancer,” which means that the role of thoracoscopic lobectomy in the treatment of benign or early malignant lung lesions has been confirmed [8, 9].

The article "Computerized Tomography Image Features under the Reconstruction Algorithm in the Evaluation of the Effect of Ropivacaine Combined with Dexamethasone and Dexmedetomidine on Assisted Thoracoscopic Lobectomy" was published in 2021. Journal: J Healthc Eng.

With the continuous breakthrough of medical imaging technology, the revolution of life science is promoted, such as CT, which provides great help for doctors' clinical diagnosis and treatment [10]. CT is widely used in the diagnosis of lung and other lesions due to its advantages of nonoverlapping cross-sectional imaging, high density resolution, and easy detection of small lesions, as well as energy spectrum and perfusion functional imaging [11, 12]. However, the current segmentation of conventional CT images has great limitations and challenges, and there are problems such as blurred boundary of lesions and insignificant brightness difference [13, 14]. Image reconstruction technology plays an important role in many fields. In the research and implementation of reconstruction algorithms, there are a series of extremely complex image processing and mathematical calculation problems [15, 16]. The essence of backprojection reconstruction refers to evenly erasing (backprojection) the ray projection from the finite object space onto all points in the infinite space reached by the ray, including the original pixel value of 0 points. At present, algorithms such as image reconstruction and computer-assisted medical image analysis have obvious advantages in major breakthroughs in technology and improvement of the medical level and have also become an effective way to solve medical image problems [17].

The article "Computerized Tomography Image Features under the Reconstruction Algorithm in the Evaluation of the Effect of Ropivacaine Combined with Dexamethasone and Dexmedetomidine on Assisted Thoracoscopic Lobectomy" was published in 2021. Journal: J Healthc Eng.

Therefore, it was attempted to construct a filtering backprojection reconstruction algorithm. The ramp-Lak filter was convolved with sin(*x*)/*x* to obtain the Shepp-Logan filter. Reconstruction of CT images and noisy data was carried out through the sheep-Logan filter to evaluate the effect of ropivacaine combined with dexamethasone and dexmedetomidine on assisted thoracoscopic lobectomy using CT image features based on reconstruction algorithm.

## 2. Materials and Methods

### 2.1. The General Information

In this study, 110 patients undergoing laparoscopy-guided lobectomy admitted to the hospital from January 2019 to September 2020 were collected as the research objects. There were 58 male patients and 52 female patients, aged 52.37 ± 5.68 years. The study had been approved by the Ethics Committee of the hospital. Patients and their families understood the content and methods of the study and signed corresponding informed consent forms.

The inclusion criteria were as follows: (i) patients who underwent lobectomy after prepathological and imaging diagnosis of lobectomy; (ii) patients aged between 45 and 65 years old; (iii) patients without metastasis of lung lesions, mediastinal lymph node enlargement, or pleural hypertrophy occurred; (iv) patients who were not recently treated with other drugs or antibiotics in the study; (v) patients with normal coagulation function and platelets.

The exclusion criteria were as follows: (i) patients with other systemic or organ lesions; (ii) patients who did not cooperate with treatment due to personal or other factors; (iii) patients with incomplete clinical data and medical history.

### 2.2. Anesthesia and Surgical Methods of Patients

All patients were fasting and abstaining from drinking six hours before anesthesia induction, and all vital signs including heart rate, diastolic blood pressure, systolic blood pressure, pulse oxygen saturation, and mean arterial pressure were monitored before surgery. 0.5% ropivacaine combined with 30 mL 1 *μ*g/Kg DEX was used. Routine disinfection and towel laying were performed on the surgical position, nerve block was performed under ultrasound guidance, and puncture was performed after local anesthesia with 1% lidocaine at the puncture site. After puncture to the specified location, local anesthesia was injected, and two-point blocking method was adopted according to the intercostal space of the surgical incision.

10 mL of drugs was injected into each puncture site, and a mixture of 0.5% ropivacaine and 1 *μ*g/Kg DEX was used as an anesthetic. The nerve block results were tested with alcohol cotton balls ten minutes after the injection.

The article "Computerized Tomography Image Features under the Reconstruction Algorithm in the Evaluation of the Effect of Ropivacaine Combined with Dexamethasone and Dexmedetomidine on Assisted Thoracoscopic Lobectomy" was published in 2021. Journal: J Healthc Eng.

The lobectomy incision was made between the midaxillary line and the front of the axillary line in the fifth intercostal area, which was close to the hilum at a small angle to facilitate the operation of hand instruments along the longitudinal axis. Hemodynamic indexes of patients were monitored in real time during surgery, and corresponding vasoactive drugs were used to correct intraoperative hemodynamic instability.

All patients enrolled in the study underwent chest enhanced CT scans, which were interpreted by two attending physicians or radiologists with extensive clinical experience. If there was a difference between the two, a third physician should be asked to interpret. CT was used to observe and analyze the specific location of lung lesions, the maximum diameter of the lesion site, and hilar and mediastinal lymph node enlargement.

### 2.3. Backprojection Reconstruction Algorithm

When the backprojection reconstruction algorithm processes medical image data, the processed image is regarded as a two-dimensional matrix *x*. The image reconstruction process is as shown in the following equation:

(1) $$\begin{array}{c} T_{\left(x\right)}=d\left(\sum_{n=1}^{y}H_{x}+p\right). \end{array}$$

In equation (1), *T*_(*x*)_ is the feature map obtained by weighting the image matrix by the convolution kernel, *H* represents the convolution kernel, *p* is the bias, *n* is the square of the size of the convolution kernel, and *d* represents the activation function. The backpropagation algorithm can accurately identify the optimal parameters in the network during the process of training the neural network. It is currently commonly used and effective. The update rule of each layer of convolution kernel *H* is as shown in the following equation:

(2) $$\begin{array}{c} H_{\alpha +1}=H_{\alpha }+\Delta H_{\alpha +1}, \end{array}$$

(3) $$\begin{array}{c} \Delta H_{\alpha +1}=\beta H_{\alpha }-\theta \sigma \nabla aH_{\alpha }. \end{array}$$

In equations (2) and (3), *H* is the convolution kernel, *α* is the number of layers, *β* is the weight of the gradient value of the previous layer, *δ* is the learning factor, *θ* is the momentum, and *a* is the loss function. The medical image reconstruction process based on backprojection is shown in Figure 1.

The network parameters are adjusted by backpropagation by minimizing the residuals of the reconstructed image and the corresponding real image, as shown in Figure 1, which is the network training process. The optimized network is obtained by training, and the aliased image is input in it to perform image reconstruction so that the obtained high-quality images can be used in clinical medical diagnosis.

The article "Computerized Tomography Image Features under the Reconstruction Algorithm in the Evaluation of the Effect of Ropivacaine Combined with Dexamethasone and Dexmedetomidine on Assisted Thoracoscopic Lobectomy" was published in 2021. Journal: J Healthc Eng.

Neural networks have independent connection and calculation methods, but they are all based on backpropagation algorithms, on which network parameters are adjusted and optimized.

(4) $$\begin{array}{c} T\left(n\right)=\int_{-\infty }^{+\infty }I\left(x\right)O\left(n-x\right)Y_{x}. \end{array}$$

It is supposed that *f*(*a*, *b*) is the image to be reconstructed, *T*(*s*, *α*) denotes a parallel projection of *f*(*a*, *b*) acquired at an angle, and *c* is the coordinate axis of the projected X-ray parallel to the angle *α*. The coordinate axis is perpendicular to the coordinate axis where *S* is located; then, there is the following equation:

(5) $$\begin{array}{c} T\left(s,\alpha \right)=\int_{-\infty }^{+\infty }f\left(s,c\right)\text{d}s. \end{array}$$

In equation (5), *s* represents the distance from the projected ray to the center of symmetry (i.e., the center of rotation). One-dimensional Fourier transform is performed on *T*(*s*, *α*) of equation (5).

(6) $$\begin{array}{c} T\left(\varpi ,\alpha \right)=\int_{-\infty }^{+\infty }T\left(s,\alpha \right)e^{-2jn\varpi s}\text{d}t. \end{array}$$

Equation (1) is substituted into equation (2) to get the following equation:

(7) $$\begin{array}{c} T\left(\varpi ,\alpha \right)=\int_{-\infty }^{+\infty }\int_{-\infty }^{+\infty }f\left(s,c\right)e^{-2jn\varpi s}\text{d}t\text{d}s. \end{array}$$

In equation (7), *ω* represents the filter function, *c* is the coordinate axis parallel to the projected X-ray under the angle *α*, and *s* represents the distance from the projected ray to the center of symmetry (i.e., the center of rotation).  Figure 2 shows the reconstructed image space coordinate system and projection space coordinate system.

In Figure 2, the coordinates of point *n* in the *a*-*o*-*b* coordinate system are shown in equations (8) and (9).

(8) $$\begin{array}{c} a=R\;\cos\beta , \end{array}$$

(9) $$\begin{array}{c} b=R\;\sin\beta . \end{array}$$

In the equations, *R* represents the distance between the point *n* and the origin in Figure 2. Similarly, the coordinates of point *n* in *s*-*o*-*c* are shown in equations (10)–(13).

(10) $$\begin{array}{c} s=R\;\cos\left(\beta -\alpha \right), \end{array}$$

(11) $$\begin{array}{c} R\;\cos\left(\beta -\alpha \right)=a\;\cos\;\alpha +b\;\sin\;\alpha , \end{array}$$

(12) $$\begin{array}{c} c=R\;\sin\left(\beta -\alpha \right), \end{array}$$

(13) $$\begin{array}{c} R\;\sin\left(\beta -\alpha \right)=b\;\cos\;\alpha +a\;\sin\;\alpha . \end{array}$$

*R* represents the distance between the point *n* and the origin in Figure 2. The above equations are substituted into equation (7) to get the following equation:

(14) $$\begin{array}{c} T\left(\varpi ,\alpha \right)=\int_{-\infty }^{+\infty }\int_{-\infty }^{+\infty }f\left(a,b\right)e^{-2jn\varpi \left(a\;\cos\;\alpha +b\;\sin\;\alpha \right)}\text{d}a\text{d}b. \end{array}$$

The two-dimensional Fourier transform of the image *f*(*a*, *b*) to be reconstructed is set as *F*(*i*, *j*); then, *F*(*i*, *j*) is expressed as follows:

(15) $$\begin{array}{c} F\left(i,j\right)=\int_{-\infty }^{+\infty }\int_{-\infty }^{+\infty }f\left(a,b\right)e^{-2jn\left(ia+jb\right)}\text{d}a\text{d}b. \end{array}$$

It is supposed that equations (16) and (17) are true.

(16) $$\begin{array}{c} i=\varpi \;\cos\;\alpha , \end{array}$$

(17) $$\begin{array}{c} j=\varpi \;\sin\;\alpha . \end{array}$$

Then, there is the following equation:

(18) $$\begin{array}{c} F\left(\varpi \;\cos\;a,\varpi \;\sin\;a\right)=T\left(\varpi ,a\right). \end{array}$$

According to the Fourier transform, the image function *f*(*a*, *b*) can be restored by its inverse Fourier transform *F*(*i*, *j*).

(19) $$\begin{array}{c} f\left(a,b\right)=\int_{-\infty }^{+\infty }\int_{-\infty }^{+\infty }F\left(i,j\right)e^{2jn\left(ia+jb\right)}\text{d}i\text{d}j. \end{array}$$

*i*=*ϖ*  cos  *α* and *j*=*ϖ*  sin  *α*; then, there is equation (20) after the calculation of equation (18).

(20) $$\begin{array}{c} f\left(a,b\right)=\int_{0}^{2n}\int_{-\infty }^{+\infty }T\left(\varpi ,a\right)e^{j2n\varpi \left(a\;\cos\;\alpha +b\;\sin\;\alpha \right)}\varpi \text{d}\varpi \text{d}\theta . \end{array}$$

Equation (19) is transformed into the following form using symmetric relationship (21), as shown in equation (22).

(21) $$\begin{array}{c} T\left(\varpi ,\alpha +\pi \right)=T\left(-\varpi ,\alpha \right), \end{array}$$

(22) $$\begin{array}{c} f\left(a,b\right)=\int_{0}^{\pi }\text{d}\alpha \int_{-\infty }^{+\infty }T\left(\varpi ,a\right)\left|\varpi \right|e^{j2n\varpi \left(a\;\cos\;\alpha +b\;\sin\;\alpha \right)}\text{d}\varpi , \end{array}$$

(23) $$\begin{array}{c} g\left(a\;\cos\;\alpha +b\;\sin\;\alpha \right)=\int_{-\infty }^{+\infty }T\left(\varpi ,a\right)\left|\varpi \right|e^{j2n\varpi \left(a\;\cos\;\alpha +b\;\sin\;\alpha \right)}\text{d}\varpi , \end{array}$$

(24) $$\begin{array}{c} f\left(a,b\right)=\int_{0}^{\pi }g\left(a\;\cos\;\alpha +b\;\sin\;\alpha \right)\text{d}\alpha . \end{array}$$

Equations (23) and (24) are the main equations for filtering backprojection, |*ω*| in (22) represents the filter function, and *f*(*a*, *b*) is the reconstructed image.

The article "Computerized Tomography Image Features under the Reconstruction Algorithm in the Evaluation of the Effect of Ropivacaine Combined with Dexamethasone and Dexmedetomidine on Assisted Thoracoscopic Lobectomy" was published in 2021. Journal: J Healthc Eng.

### 2.4. Image Reconstruction and Effect Evaluation

In this study, a backprojection image reconstruction algorithm was used to reconstruct the lung lesions of patients undergoing lobectomy, and filtering function was added to solve the problem of image sharpness. In addition, the iterative reconstruction algorithm (using the method of solving linear equations to reconstruct the image) and Fourier transform analytical method were introduced. In the arterial phase of chest enhanced CT, the pulmonary artery, pulmonary vein, lesion, and blood-supplying artery were reconstructed. Through the reconstruction of 3D images, the lesions were presented more clearly in the form of three dimensions and visualization, so as to realize the simulation effect.

### 2.5. Statistical Methods

SPSS 19.0 was employed for data statistics and analysis. Mean ± standard deviation (-*x* ± *s*) was how measurement data were expressed, and percentage was how count data were expressed. The pairwise comparison was performed by analysis of variance. The difference was statistically considerable with *P* < 0.05.

## 3. Results

### 3.1. Running Time of the CT Image Reconstruction Algorithm

Figure 3 shows the running time of CT image reconstruction by Fourier transform analysis, iterative reconstruction algorithm, and backprojection image reconstruction algorithm. Figures 3(a) and 3(b) show the calculation time under different block and different overlap step parameter settings, respectively. The Fourier transform analysis had the shortest running time when the overlap step was 8, the block size was 32 × 32, and the overlap step was 16. The iterative reconstruction algorithm had the shortest running time when the overlap step was 16 and the block size was 48 × 48. When the overlap step was 16 and the block size was 32 × 32, the backprojection image reconstruction algorithm had the shortest running time.

### 3.2. Analysis of the Effect of CT Image Reconstruction

According to the noise characteristics in the data, the filtering function was applied to the original data, and the signal in the image was filtered, removing noise and artifacts to reconstruct the image. In Figure 4, there were patchy, subsegmental, and segmental ground-glass density shadows in the CT images of pulmonary lesions, which were separated into paving stone-like changes by the thickening of small honeycomb-like interlobular septa. In addition, large consolidation in the middle lobe of the right lung and patchy consolidation in the posterior basal segment of the lower lobe were observed. The density shadow of ground glass and the thickening of interlobular interval were seen obviously after image removal and processing by the backprojection filter reconstruction algorithm.

The article "Computerized Tomography Image Features under the Reconstruction Algorithm in the Evaluation of the Effect of Ropivacaine Combined with Dexamethasone and Dexmedetomidine on Assisted Thoracoscopic Lobectomy" was published in 2021. Journal: J Healthc Eng.

### 3.3. Analysis of the Reconstruction Effect of Three Algorithms

Figure 5 shows the CT images of a central lung cancer patient and a right upper lobe lung cancer patient, as well as the results of reconstruction by Fourier transform analysis, iterative reconstruction algorithm, and backprojection image reconstruction algorithm. Through adaptive image selection and super-resolution reconstruction, the backprojection reconstruction algorithm continuously corrected the structural information of the target image block, so as to obtain high definition and clear image edge. High-resolution images with dramatically enhanced details can eliminate the interference of image noise and artifacts and reconstruct clear CT images. The image clarity and resolution obtained by the backprojection reconstruction algorithm were superior to those of Fourier transform analysis and iterative reconstruction algorithm.

### 3.4. Detection Rate of Pulmonary Nodules by Three Reconstruction Algorithms

Figure 6 shows the comparison of the detection rates of pulmonary nodules of different sizes after the three algorithms, namely, Fourier transform analysis method, iterative reconstruction algorithm, and backprojection image reconstruction, processed the lung CT images. For pulmonary nodules smaller than 6 mm, the detection rates of the three algorithms were 90.98%, 87.53%, and 92.35%, respectively. For 6–30 mm lung nodules, the detection rates of the three algorithms were 88.32%, 90.87%, and 95.44%, respectively. The detection rate of pulmonary nodules of different sizes by backprojection image reconstruction algorithm was significantly higher than that by the Fourier transform analytical method and iterative reconstruction algorithm (*P* < 0.05).

### 3.5. Patient's Lung Disease Types

Figure 7 shows the types of lung lesions and their proportion in patients undergoing lobectomy. Patients with central lung tumors and right upper lobe tumors accounted for a relatively high proportion of 43.21% and 29.54%, respectively, followed by tuberculosis, severe lung infection, and pulmonary fibrosis, accounting for 8.11%, 8.93%, and 10.21%, respectively.

### 3.6. VAS Scores of Patients at Different Postoperative Periods

Figure 8 shows the VAS scores at different periods after thoracoscopic lobectomy.  Figure 8(a) shows the VAS score under the resting state, and Figure 8(b) shows the VAS score under the exercise state. Ropivacaine combined with dexamethasone and dexmedetomidine was used for anesthesia induction and lobectomy after nerve block, and VAS scores decreased with the extension of postoperative time. The VAS score decreased to a low level after five days.

The article "Computerized Tomography Image Features under the Reconstruction Algorithm in the Evaluation of the Effect of Ropivacaine Combined with Dexamethasone and Dexmedetomidine on Assisted Thoracoscopic Lobectomy" was published in 2021. Journal: J Healthc Eng.

## 4. Discussion

The basis of CT image reconstruction is as follows. The same X-ray intensity passes through different substances, and different substances in the human body are distinguished by using this law [18, 19]. The structures that X-rays pass through each layer of the body in a CT scan are broken up into small cubes called voxels. Each cube corresponds to a separate attenuation signal, and this signal is fed into the corresponding cell in the image plane matrix called pixel. The attenuation signal of each voxel is input into the corresponding pixel and then reflected in different gray scales, which is the process of CT image reconstruction [20, 21]. For the backprojection image reconstruction algorithm, the problem of image sharpness is solved by adding a filter function. The reconstructed image is blurred when the filter function is not added, and the reconstructed image after the filter function is added can make it clear. Due to the fast reconstruction speed and high image quality of the backprojection filter, it has become the most commonly used CT image reconstruction method. Although the iterative reconstruction algorithm has been proposed very early, due to its large amount of calculation and slow reconstruction speed, it depends on the breakthrough of computer performance. Therefore, the backprojection reconstruction algorithm is widely used in current applications [22, 23]. In this study, a backprojection image reconstruction algorithm was used to reconstruct the lung lesions of patients undergoing lobectomy by CT three-dimensional reconstruction, and a filter function was added to solve the problem of image sharpness. In addition, iterative reconstruction algorithm and Fourier transform analysis method were introduced. Aiming at the arterial phase of enhanced CT of the patient's chest, the pulmonary artery, pulmonary vein, lesion, and blood supply artery were reconstructed, and the lesion was visualized more clearly through the reconstructed three-dimensional image, achieving the effect of simulation.

Through the backprojection reconstruction algorithm to process the CT image, it was found that when the overlap step was 16 and the block size was 32 × 32, the backprojection image reconstruction algorithm had the shortest running time. Therefore, to ensure that a higher-quality image was obtained after reconstruction, the setting of image block parameters should not affect the reconstruction result. The image separation parameters of this study were set as follows. The block size was 32 × 32, and the overlap step length was 16 pixels. The detection rate of backprojection image reconstruction algorithm for lung nodules smaller than 6 mm and 6–30 mm was significantly higher than that of the Fourier transform analytical method and iterative reconstruction algorithm (*P* < 0.05). The results were similar to those of Yoshida et al. [24], which showed that the backprojection image reconstruction algorithm can continuously modify the structure information of the target image through super-resolution reconstruction, make the image clear, and facilitate the identification of the lesion. The patients included in this study were treated with ropivacaine combined with dexamethasone and dexmedetomidine for induction of anesthesia and lobectomy for nerve block. The patient's VAS score decreased with the extension of postoperative time. After five days, the patient's VAS score can be reduced to a lower level. This was similar to the results of Williams et al. [25]. It was verified that combined induction of anesthesia and nerve block had a positive effect on postoperative pain and postoperative recovery.

The article "Computerized Tomography Image Features under the Reconstruction Algorithm in the Evaluation of the Effect of Ropivacaine Combined with Dexamethasone and Dexmedetomidine on Assisted Thoracoscopic Lobectomy" was published in 2021. Journal: J Healthc Eng.

## 5. Conclusion

In this study, a backprojection image reconstruction algorithm was established and applied to CT images of patients undergoing thoracoscopic lobectomy. The image was reconstructed to remove noise and artifacts to obtain a clear image and identify lesions. Then, the effect of ropivacaine combined with DXM and DEX in blocking thoracoscopic lobectomy was studied by evaluating CT image features based on reconstruction algorithm. The results showed that ropivacaine combined with dexamethasone and dexmedetomidine had ideal sedation and analgesia effects in patients with thoracoscopic lobectomy. The CT image based on the backprojection reconstruction algorithm had a high recognition accuracy for lung lesions, which was worth applying to clinical diagnosis. However, this study lacked comparison with other intelligent algorithms and was less representative. Therefore, this aspect will be improved and optimized in the subsequent experiments, and the CT image features based on reconstruction algorithm will be further analyzed to evaluate the effect of ropivacaine combined with dexamethasone and dexmedetomidine in the treatment of video-assisted thoracoscopic lobectomy. In conclusion, this study provides a reference for the application of intelligent reconstruction algorithms such as backprojection filtering in medical images.

## Figures and Tables

**Figure 1:** Medical image reconstruction (a) and reconstruction effect (b) based on backprojection.

**Figure 2:** Image space coordinate system and projection space coordinate system.

The article "Computerized Tomography Image Features under the Reconstruction Algorithm in the Evaluation of the Effect of Ropivacaine Combined with Dexamethasone and Dexmedetomidine on Assisted Thoracoscopic Lobectomy" was published in 2021. Journal: J Healthc Eng.

**Figure 3:** Image reconstruction running time. (a) The running time of different overlapping steps. (b) The running time of different block sizes.

**Figure 4:** Reconstruction of CT images of lungs by backprojection.

**Figure 5:** Analysis of the reconstruction effect of the three algorithms.

**Figure 6:** Detection rates of pulmonary nodules by three reconstruction algorithms.

**Figure 7:** Types of lung lesions in the patients.

**Figure 8:** VAS score of patients after operation. (a) The VAS score in the resting state. (b) The VAS score in the exercise state.

## Data Availability

The data used to support the findings of this study are available from the corresponding author upon request.
